This article has been retracted.

# RNA Interference Targeting Slug Increases Cholangiocarcinoma Cell Sensitivity to Cisplatin via Upregulating PUMA

**DOI:** 10.3390/ijms12010385

**Published:** 2011-01-14

**Authors:** Kejun Zhang, Dong Chen, Xingang Wang, Shaoyan Zhang, Jigang Wang, Yuan Gao, Bomin Yan

**Affiliations:** 1 General Surgery of the Affiliated Hospital of Medical College, Qingdao University, Qingdao, Shan Dong Province 266003, China; E-Mails: wlsdermyy@163.com (K.Z); wangxingang77521@126.com (X.W.); yanbm818@yahoo.com.cn (B.Y.); 2 Laboratory of the Affiliated Hospital of Medical College, Qingdao University, Qingdao, Shan Dong Province 266003, China; E-Mail: zlfzyj2009@163.com; 3 Pathology, The Affiliated Hospital of Medical College, QingDao University, Qingdao, Shan Dong Province 266003, China; E-Mail: Love5028@sohu.com; 4 Molecular Biology, The Affiliated Hospital of Medical College, QingDao University, Qingdao, Shan Dong Province 266003, China; E-Mail: isgs@rocketmail.com

**Keywords:** cisplatin, chemotherapy, slug, PUMA, E-cadherin

## Abstract

Slug is an E-cadherin repressor and a suppressor of PUMA (p53 upregulated modulator of apoptosis) and it has recently been demonstrated that Slug plays an important role in controlling apoptosis. In this study, we examined whether Slug’s ability to silence expression suppresses the growth of cholangiocarcinoma cells and/or sensitizes cholangiocarcinoma cells to chemotherapeutic agents through induction of apoptosis. We targeted the Slug gene using siRNA (Slug siRNA) via full Slug cDNA plasmid (Slug cDNA) transfection of cholangiocarcinoma cells. Slug siRNA, cisplatin, or Slug siRNA in combination with cisplatin, were used to treat cholangiocarcinoma cells *in vitro*. Western blot was used to detect the expression of Slug, PUMA, and E-cadherin protein. TUNEL, Annexin V Staining, and cell cycle analysis were used to detect apoptosis. A nude mice subcutaneous xenograft model of QBC939 cells was used to assess the effect of Slug silencing and/or cisplatin on tumor growth. Immunohistochemical staining was used to analyze the expression of Slug and PUMA. TUNEL was used to detect apoptosis *in vivo*. The results showed that PUMA and E-cadherin expression in cholangiocarcinoma cells is Slug dependent. We demonstrated that Slug silencing and cisplatin both promote apoptosis by upregulation of PUMA, not by upregulation of E-cadherin. Slug silencing significantly sensitized cholangiocarcinoma cells to **c**isplatin through upregulation of PUMA. Finally, we showed that Slug silencing suppressed the growth of QBC939 xenograft tumors and sensitized the tumor cells to cisplatin through PUMA upregulation and induction of apoptosis. Our findings indicate that Slug is an important modulator of the therapeutic response of cholangiocarcinoma cells and is potentially useful as a sensitizer in cholangiocarcinoma therapy. One of the mechanisms is the regulation of PUMA by Slug.

## 1. Introduction

Despite the aggressive multidisciplinary cancer therapies that have been used clinically, the prognosis of cholangiocarcinoma patients is extremely poor due to the low resection rate and the tolerance of the cancer to chemotherapy and radiotherapy [1,2]. For this reason, it is important to find new methods to enhance the sensitivity of cholangiocarcinoma cells to chemotherapeutic agents. Gene therapy for cholangiocarcinoma is potentially a promising approach. The identification of molecules involved in the regulation and induction of apoptosis in cholangiocarcinoma has recently been reported and has generated new biological treatments aimed at enhancing chemotherapy-induced cell apoptosis [3–5].

The human Slug gene belongs to the highly conserved Slug/Snail family of transcription repressors, master regulators of neural crest cell specification and melanocyte migration during development in vertebrates [6–10]. Previous studies have demonstrated that the overexpression of Slug can be found in many kinds of cancer [11–14]. Moreover, Slug activates multiple signal intermediates, such as E-cadherin, which are key factors that influence the events of tumor invasion and metastasis [15,16]. In addition, Slug promotes survival and hinders cell death by directly suppressing PUMA, a key BH3-only antagonist of the anti-apoptotic Bcl-2 protein [17,18]. A previous study has demonstrated that PUMA is an important modulator of the therapeutic response of lung cancer cells and is potentially useful as a sensitizer in lung cancer therapy [19]. There have been a few studies devoted to the role of Slug in the chemoresistance of cancer cells to anti-cancer agents. A recent report indicated the possibility that Slug enhances chemoresistance of malignant mesothelioma cells to doxorubicin, paclitaxel, and vincristine [20]. It has been reported by Kurrey NK that Slug plays a critical role in the ability of a cancer cell to acquire stem cell characteristics to resist radiotherapy or chemotherapy-mediated cellular stress [21]. Roberta *et al*. [22] has reported that Slug down-regulation facilitates the apoptosis induced by proapoptotic drugs in neuroblastoma cells and decreases their invasion capability *in vitro* and *in vivo*, and that Slug silencing enhances the efficacy of cisplatin and fotemustine in the treatment of melanoma [23].

However, to the best of our knowledge, the roles and possible mechanisms of Slug in the chemoresistance of cholangiocarcinoma cells to cisplatin have not been previously reported. The aim of this study is to investigate and define the ability and mechanism of Slug silencing to increase the susceptibility of cholangiocarcinoma cell lines to the currently used cytotoxic drug cisplatin.

## 2. Materials and Methods

### 2.1. Cell Culture

The human cholangiocarcinoma cell lines QBC939, RBE, ICC-9810 and FRH 0201 were purchased from ATCC and conserved in the central laboratory of the first affiliated Hospital of Suzhou University, China. Cells were grown in HAMs F12 medium supplemented with 10% fetal bovine serum at 37 °C in a 5% CO_2_ humidified atmosphere.

### 2.2. siRNA and cDNA Transfection

The siRNA targeting Slug (Slug siRNA, sc-38393) and mock siRNA (mock, sc-37007), the siRNA targeting PUMA (PUMA siRNA, sc-37153) and mock siRNA (mock, sc-33007) was obtained from Santa Cruz Biotechnology. Mock siRNA is a non-targeting 0–25nt siRNA designed to serve as a negative control. In a six well tissue culture plate, we seeded 2 × 10^5^ cholangiocarcinoma cells per well in 2 mL antibiotic-free normal growth medium supplemented with FBS. We then incubated the QBC939 cells at 37 °C in a CO_2_ incubator until the cells were 60–80% confluent for 24 hours. The following solutions were prepared: Solution A: For each transfection, 2–8 μL of siRNA duplex (*i.e.*, 0.25–1 μg siRNA) was diluted into 100 μL siRNA transfection medium: sc-36868 (Santa Cruz). Solution B: For each transfection, 6 μL of siRNA transfection reagent: sc-29528 (Santa Cruz, CA, USA) was diluted into 100 μL siRNA transfection medium: sc-36868(Santa Cruz, CA, USA). The siRNA duplex solution was then added (Solution A) directly to the diluted transfection reagent (Solution B) using a pipette and mixed gently by pipetting the solution up and down, then incubated for 30 minutes at room temperature. We then washed the cells once with 2 mL of siRNA transfection medium: sc-36868. For each transfection, we added 0.8 mL siRNA transfection medium to each tube containing the siRNA transfection reagent mixture (Solution A + Solution B) and then mixed gently and overlayed the mixture onto the washed cells. The cells were then incubated for 6 hours at 37 °C in a CO_2_ incubator. A volume of 1 mL of normal growth medium containing 2 times the normal serum and antibiotics concentration (2 × normal growth medium) was then added without removing the transfection mixture, and the cells were subsequently incubated for an additional 24 hours, at which time the medium was aspirated and we proceeded immediately to the next step. We performed Western blot on the cells 0–72 h after the addition of fresh medium in the step above. Mock siRNA containing a scrambled sequence that would not lead to the specific degradation of cellular Slug mRNA was transfected as above. The plasmid vector with the full coding region of human Slug (pcDNA3-Slug cDNA, Slug cDNA in brief) and the mock vector (pcDNA3-EGFP, mock cDNA in brief) were created in our laboratory (16). Transfection of Slug cDNA was performed using Lipofectamine 2000 (Invitrogen, Carlsbad, CA, USA) according to the manufacturer’s instructions. In brief, 1 μg Slug cDNA was mixed with 3 μg Lipofectamine 2000 at a final concentration of 2 μg Slug cDNA/mL dissolved in OPTI-MEM I (Invitrogen), and the resulting complex was added to the cells and the FRH 0201cells were incubated with the complex for 4 h. FRH 0201 cells were washed with PBS and further incubated with the culture medium for specified time periods ranging from 0–72 h. Stably expressed Slug siRNA (mock) clones were selected by using medium containing G418 (500 μg/mL) for 28 days. Cells were routinely maintained in selection media containing 200 μg/mL of G418-sulfate to avoid overgrowth of nontransfected cells.

### 2.3. Western Blot

We collected approximately 2.0 × 10^7^ cells (at different conditions) by low-speed centrifugation (e.g., 200 × g) at room temperature for 5 minutes and carefully removed the culture medium. Next, we washed the pellet with PBS at room temperature, and again collected cells by low-speed centrifugation and carefully removed the supernatant. We added 1.0 mL of ice cold RIPA buffer with freshly added Protease Inhibitors and gently resuspended the cells in RIPA buffer with a pipette and incubated the cells on ice for 30 minutes. We then further disrupted and homogenized the cells by hydrodynamic shearing (21-gauge needle), dounce homogenization (Optional: Add 10 μL of 10 mg/mL PMSF stock), and then incubated the cells for 30 minutes on ice. Next, samples were transfered to microcentrifuge tube(s) and centrifuged at 10,000 × g for 10 minutes at 4 °C. The supernatant fluid represented the total cell lysate and the supernatant was transferred to a new microfuge tube and represented the whole cell lysate. Total protein was measured in the extract by the Bradford assay. Primary antibodies were as follows: Anti-Slug (1:200 dilution), Anti–PUMA (1:400 dilution), and Anti-ß-actin (1:500 dilution), all from Santa Cruz Biotechnology. The membrane was probed using horseradish peroxidase–conjugated immunoglobulins (DAKO) as described previously (24). Western blot images were captured using an Epi Chemi II Darkroom and Sensicam imager with Labworks 4 software (UVP).

### 2.4. Terminal Deoxynucleotidyl Transferase Biotin-dUTP Nick End Labeling Assay

Cells in different groups were cultured on chamber slides for 24 h. Apoptosis of the cells was evaluated on the basis of the TUNEL assay using the Dead End Fluorometric TUNEL System (Promega, Madison, WI, USA) according to the manufacturer’s instructions. All assays were performed in quadruplicate.

### 2.5. Cell Cycle Analysis

The cells in different groups and time points were washed twice with PBS and fixed with 70% ethanol/PBS. They were then treated with 0. 5 mg/mL RNase (Sigma) in PBS with 0.1% saponin, and incubated at 37 °C for 30 min before staining with 20 μg/mL PI for 30 min at 4 °C. The cells (1 × 10^6^) were then analyzed for DNA content using a FACSCalibur flow cytometer equipped with CellQuest software (Becton Dickinson Immunocytometry Systems).

### 2.6. Annexin V Staining

The Annexin V assays were performed according to the manufacture’s protocol (PharMingen). Briefly, the cultured cells were collected, washed with binding buffer, and incubated in 200 μL of a binding buffer containing 5 μL of Annexin-V-FITC. The nuclei were counterstained with PI. The percentage of apoptotic cells was determined using a FACSCalibur flow cytometer (Becton Dickinson Immunocytometry Systems, San Jose, CA, USA).

### 2.7. Xenograft Tumors

Immunodeficient female mice, 4 to 6 weeks old, were purchased from the Shanghai Animal Center. Autoclaved cages containing food and water were changed once a week. Mouse body weight was measured every 3 to 4 days. On the day of tumor cell inoculation, tumor cells at 70% to 80% confluence were trypsinized and resuspended in fetal bovine serum-free culture medium. Xenograft tumors were established by subcutaneous injection of 5 × 10^6^ BQC939 cells (stable transfected with Slug siRNA or mock) into the flanks of 4 to 6 week old female Nude mice (n = 6 per group). In the combination model, cisplatin (3 mg/kg/d) was injected intraperitoneally into the mice on days 6–8. Mock transfected BQC939 cells were injected into separate tumors in the same animals. Tumor growth was monitored every other day with calipers for 28 days to calculate tumor volume according to the formula [length × width^2^]/2.

### 2.8. Immunohistochemistry in Xenograft Tumors

Tumor samples fixed in 10% neutral buffered formalin were embedded in paraffin using automatic embedding equipment, after which 5 μm sections were prepared. Immunohistochemical analyses for Slug and PUMA were performed on paraffin-embedded sections of mice treated with Slug siRNA or mock siRNA according to the manufacturer’s instruction.

### 2.9. TUNEL Staining *in Vivo*

Paraffin-embedded tumor sections were used to identify apoptotic cells by terminal deoxynucleotidyl transferase-mediated dUTP nick end labeling (TUNEL) staining following the vendor’s protocol. A section was incubated with nuclease to generate DNA strand breaks for positive control. Endogenous peroxidase activity was quenched by 5% H_2_O_2_ (in methanol, v/v) and sections were incubated with terminal deoxynucleotidyl transferase labeling buffer followed with terminal deoxynucleotidyl transferase enzyme and biotinylated nucleotides (for negative control, labeling buffer was used instead of terminal deoxynucleotidyl transferase enzyme). Sections were incubated with streptavidin-conjugated horseradish peroxidase followed with 3,3′-diaminobenzidine solution (Sigma) and counterstained with diluted hematoxylin. Apoptosis was evaluated by counting the TUNEL-positive cells together with the total number of cells at 5 randomly selected fields at ×400 magnification in each tumor; the data are presented as percent TUNEL-positive cells.

### 2.10. Statistics

All statistical analyses were performed using SPSS13.0 software. The results were presented as mean ± SD of three separate assays. Differences between various groups were assessed using the ANOVA or Dunnett t-test. A P value of <0.05 was considered to indicate statistical significance.

## 3. Results

### 3.1. Slug Regulates PUMA and E-Cadherin Expression in Cholangiocarcinoma Cells

Slug expression was examined in a panel of four cholangiocarcinoma cell lines QBC939, RBE, ICC-9810, and FRH0201 by Western blot. The results indicated that the cell line FRH 0201 exhibited the lowest expression level of Slug and that QBC939 exhibited the highest expression level of Slug (Figure 1A). In this regard, the cell lines FRH 0201 and QBC939 were chosen for the studies.

The cell line FRH0201 was transiently transfected with either full length human Slug cDNA vector or the mock vector for 48 h to increase the expression of Slug. The cell line QBC939 was transiently transfected with Slug siRNA for 48 h to knock down Slug. In Slug siRNA-transfected QBC939 cells, Slug expression was barely detectable compared with parental cells (Figure 1B), whereas Slug cDNA-transfected FRH 0201 cells expressed a higher level of Slug compared with parental cells (Figure 1C).

Slug is a suppressor of PUMA transcription (18). To evaluate whether Slug plays a role in the regulation of PUMA in cholangiocarcinoma cell lines, we analyzed the expression of PUMA in Slug siRNA-transfected QBC939 cells and Slug cDNA-transfected FRH 0201 cells by Western blot. In Slug siRNA-transfected QBC939 cells, PUMA was up-regulated compared with parental cells (Figure 1B). By contrast, in Slug cDNA-transfected FRH 0201, no PUMA expression was seen compared with parental cells (Figure 1C).

It has been recently reported that the Slug transcription factor directly represses E-cadherin expression in many epithelial cancers associated with epithelial-mesenchymal transitions. The reverse correlation of Slug and E-cadherin expression has been noted in many malignant cells. We found in our study that Slug siRNA-transfected QBC939 cells showed a remarkble upregulation of E-cadherin protein compared with parental cells (Figure 1B) and that a remarkable downregulation of E-cadherin protein was shown in Slug cDNA-transfected FRH 0201 cells compared with parental cells (Figure 1C). These observations provided direct evidence that Slug regulated E-cadherin and PUMA expression in human cholangiocarcinoma cells.

### 3.2. Slug Inhibition by siRNA Promotes Apoptosis in Cholangiocarcinoma Cells

It has been previously demonstrated that Slug is involved in the control of apoptosis [17]. We next hypothesized that Slug silencing may have proapoptotic effects on cholangiocarcinoma cells. To investigate this, cell apoptosis was detected in QBC93 cells transiently transfected with Slug siRNA or mock for 48h by TUNEL analysis. It showed that the apoptosis rate in Slug siRNA-transfected QBC939 cells was significantly increased compared with the control or mock-transfected QBC939 cells (*P < 0.05, Figure 2).

To explore whether Slug inhibition by RNA interference promotes apoptosis by upregulating PUMA, and not by upregulating E-cadherin**,** we examined the effects of Z-DEVD-CHO, a caspase-3 inhibitor, on the internucleosomal degradation of DNA. It showed that the treatment of QBC939 cells with the inhibitor combined with transfection of Slug siRNA for 48 h resulted in significantly decreased cell apoptosis in contrast to only Slug siRNA treated groups (Figure 2, *P < 0.05).

### 3.3. Cisplatin promotes Cholangiocarcinoma Cells Apoptosis *in Vitro*

This study demonstrated that cisplatin induced apoptosis in human cholangiocarcinoma cell lines QBC939 and FRH0201 in a concentration- and time-dependent manner. As shown in Figure 3A and Figure B, treating the cholangiocarcinoma cells with 0.1 μg/mL cisplatin for 72 h caused only a slight increase in the proportion of apoptotic cells in the two cell lines. However, increasing the cisplatin concentration (20 μg/mL) for 72 h resulted in a sharp increase in the proportion of apoptotic cells, suggesting that cell death occurred in a dose-dependent manner (compared to control, *P < 0.05, **P < 0.01, ***P < 0.001).

When the cholangiocarcinoma cells were exposed to 20 μg/mL cisplatin, the proportion of apoptotic cells increased in a time-dependent manner. Almost 70% (FRH 0201), over 40% (QBC939) of the other cell population underwent apoptosis after 72 h, compared with ≤5% of the control (BPS-treated) cells (Figure 3A,B).

Similar results were obtained when the apoptosis was monitored by cell cycle analysis. Exposure to 20 μg/mL cisplatin for 12–24 h had no remarkable effect on the cell cycle distribution of the cholangiocarcinoma cells. However, the cisplatin treatment for 48–72 h resulted in a progressive increase in the sub-G1 cell fraction. (Figure 3C, D) (contrast to control, *P < 0.05, **P < 0.01, ***P < 0.001).

### 3.4. Cisplatin Cytotoxicity Is Associated with PUMA Induction

The effects of cisplatin on the intracellular level of PUMA were analyzed to additionally examine the relationship between cell death and PUMA in the QBC939 and FRH 0201 cholangiocarcinoma cells. The cells were treated with various cisplatin concentrations for 72 h, or the cells were treated with 20 μg/mL cisplatin concentrations for various lengths of time. The PUMA and E-cadherin extracted from the cells were subjected to Western blot analysis. A representative result of QBC939 and FRH 0201 is shown in Figure 4A–D. The amount of PUMA was increased in a concentration-dependent and time-dependent manner, reaching a maximum level at 20 μg/mL of cisplatin or 72 h treatment.

The results demonstrated that cisplatin did not obviously promote or reduce E-cadherin expression (Figure 4A–D). These observations provided direct evidence that cisplatin-induced apoptosis was not E-cadherin- dependent.

To determine whether the induction of cell death in cisplatin-treated cholangiocarcinoma cells was due, in part, to regulation of PUMA expression, QBC939 and FRH 0201 cells were exposed to a cisplatin concentration of 20 μg/mL for 6 h, after which time the cisplatin-treated cells were transfected PUMA siRNA for 72 h to knock down PUMA. This study demonstrated that induction of PUMA was not shown in any of the PUMA siRNA treated sample populations (Figure 4E,F). Cisplatin combined with PUMA siRNA did not induce obvious apoptosis in QBC939 and FRH 0201 cells (Figure 4G,H, *P < 0.01). By contrast, mock-transfected cells exhibited PUMA levels or an apoptosis level similar to that found in cells treated only with cisplatin (Figure 4G,H).

### 3.5. Slug Silencing and Cisplatin Treatment Act in Concert to Induce Apoptosis in Cholangiocarcinoma Cells

Given the activity of Slug in cell survival through regulation of proapoptotic factor PUMA, and the fact that cisplatin promotes apoptosis by upregulating PUMA, we assessed the apoptosis susceptibility of Slug siRNA-transfected QBC939 cells in the presence of 5 μg/mL cisplatin for 48 h. At the end of each treatment, cells were fixed and stained for TUNEL analysis. siRNA-transfected QBC939 cells combined with 5 μg/mL cisplatin showed a significantly increased apoptosis rate compared with siRNA-transfection only or cisplatin treatment alone (*P < 0.05, **P < 0.01) (Figure 5).

### 3.6. Slug Silencing Suppresses Cholangiocarcinoma Tumor Growth and Sensitizes Cholangiocarcinoma Xenografts to Cisplatin *in Vivo*

To determine whether Slug silencing confers antitumor activity *in vivo*, established 6 × 10^6^ QBC939 cells (stable transfection with Slug siRNA or mock siRNA) were injected into the flanks of 4 to 6 week old female Nude mice (n = 6 per group). Mock siRNA had no effect on tumor growth compared to the control alone, with tumors doubling in volume in 28 days compared to Slug siRNA treatment groups (**P < 0.01; Figure 6A).

Furthermore, we analyzed the tumor sections from control, mock siRNA, and Slug siRNA groups for Slug and PUMA using immunohistochemistry. We observed significant expression levels of Slug in control and mock-treated tumor sections (Figure 6B). However, expression levels were drastically reduced in the tumor sections of mice treated with Slug siRNA. Furthermore, we observed drastically increased PUMA in Slug siRNA tumor sections (Figure 6B).

Analyzing tissue sections from tumors revealed that Slug siRNA, but not mock, significantly increased apoptosis in the tumors as assessed by TUNEL staining (Figure 6C). These data show that Slug silencing effectively inhibits the growth of Cholangiocarcinoma tumors through apoptosis induction.

Slug silencing was found to promote apoptosis by cisplatin *in vitro*. We wanted to determine whether such effects can be obtained in the QBC939 xenograft tumor model. To investigate the potential additive or synergistic effects, we used cisplatin (3 mg/kg/d for 4 days) in these experiments. Cisplatin treatment alone resulted in 20% growth inhibition compared with mock or PBS control, respectively (*P < 0.05, Figure 6A). In contrast, Slug siRNA combined with cisplatin resulted in >60% growth suppression (***P < 0.001, Figure 6A), indicating synergism. Analysis of tumor sections revealed that the Slug siRNA and cisplatin combination resulted in a significant increase in apoptosis compared with Slug siRNA or cisplatin alone (Figure 6C). These results suggest that Slug silencing enhances the therapeutic response of QBC939 tumors to cisplatin through apoptosis induction.

## 4. Discussion

Resistance of cholangiocarcinoma to chemotherapy is a major problem in cancer treatment [27–29]. Currently, it is generally acknowledged that chemotherapeutic agents exert their cytotoxic effects through the activation of apoptosis and promotion of apoptosis can increase the chemosensitivity of cancer cells [30,31]. For this reason, inhibited expression of some specific genes that inhibit apoptotic cell death can cause malignant cells to be relatively sensitive to the cytotoxic effect of chemotherapeutic agents.

The appearance of novel strategies for cancer treatment is based on the selective downregulation of specific targets involved in neoplastic progression. Slug seems to be a relevant target for such therapeutic intervention. Slug is detectable in many types of cancer, and its presence has been associated with poor prognosis in many malignant tumors [32–35]. Not only is Slug an inducer of epithelial-mesenchymal transition (EMT) and cell movement, it is also considered to be a factor favoring cell survival [16]. Previous studies have demonstrated that Slug overexpression exhibits a radioprotective function in TK6 cells demonstrating that it has potential as a candidate for gene therapeutic radioprotection of normal tissues [36]. Mancini *et al*. [37] has demonstrated that Slug overexpression contributes to apoptosis resistance in leukemic progenitors. Manuela Mancini reported that Slug overexpression was involved in prolonged survival and imatinib(IM)resistance of Chronic myelogenous leukemia(CML) progenitors [37]. In this report, we demonstrated for the first time that Slug silencing could efficiently promote apoptosis in cholangiocarcinoma cells. Annexin-V/PI and TUNEL staining revealed that apoptotic cell death was abundant in cells with slug repression, but almost completely absent in cells transfected with mock-siRNA. These data demonstrate that the Slug silencing gene facilitates apoptosis.

Slug, a highly conserved zinc finger transcriptional repressor, has been reported to antagonize apoptosis of hematopoietic progenitor cells by repressing PUMA transactivation [18]. In another study, it was demonstrated that suppression of the Slug gene facilitates apoptosis of fibroblast-like synoviocytes (FLS) by increasing PUMA transactivation [38].

Our current findings show that when Slug was knocked down in the QBC939 cells, the PUMA and E-cadherin proteins were upregulated in the cells with the Slug supression. When caspase-3, a downstream gene induced by upregulation of PUMA, was blocked, the cell apoptosis caused by Slug silencing was reduced. These data demonstrate that Slug silencing facilitates apoptosis by PUMA upregulation, and not by E-cadherin upregulation.

Recent studies have demonstrated that Slug silencing increases sensitivity to apoptosis induced by cisplatin, fotemustine, imatinib mesylate, etoposide, or doxorubicin [39,40]. Our study demonstrated that Slug silencing markedly enhances cisplatin-induced apoptosis in cholangiocarcinoma cells *in vivo* and *in vitro*, and that Slug overexpression could contribute to impaired apoptosis (data not shown). The mechanism by which Slug silencing induced an increase in cisplatin-induced apoptosis involves the upregulation of PUMA; moreover, Slug suppression increases the capacity of cisplatin to block the cell cycle and induce cell death and such a phenomenon is also accompanied by the upregulation of PUMA.

Previous studies have demonstrated that cisplatin-induced apoptosis in human bladder cancer cells and renal tubular cells was dependant upon PUMA [41,42]. However, Carly St has reported that cisplatin is a MAPK pathway dependent inducer of ATF3, whose expression influences cisplatin’s cytotoxic effects [43]. The mechanisms underlying the proapoptotic effect of the chemotherapeutic agent, cisplatin, are largely undefined. In the present study, we found that cisplatin caused significant induction of apoptosis of human cholangiocarcinoma cells in a time and concentration dependent manner and that this was associated with arrest of the cell cycle in G_0_-G_1_. We also found that cisplatin cytotoxicity is associated with PUMA induction, and when PUMA was suppressed the apoptosis induced by cisplatin was blocked. This suggests that an apoptosis-inducing mechanism triggered by cisplatin operates via PUMA in the cholangiocarcinoma cells. Another study, however, has found that PUMA induction by chemotherapeutic agents is abrogated in most human non-small-cell carcinoma(HNSCC)cell lines, and that cisplatin does not induce any increase in PUMA expression [44].

To investigate whether the combination of Slug knockdown and cisplatin treatment can synergistically inhibit tumor growth and increase cholangiocarcinoma cell sensitivity to cisplatin, we used a well-established Xenograft tumor model in severe combined immunodeficient mice. Slug silencing or cisplatin alone inhibited Xenograft tumor growth, and the effects of both did reach statistical significance. This result is in contrast with the findings of the *in vitro* assays. When Slug-silenced cells were treated with cisplatin, significant growth suppression and apoptosis was demonstrated.

Our results suggest that this combination of cisplatin and Slug suppression may be useful for chemoprevention and/or therapy of cholangiocarcinoma and possibly other types of cancer. Indeed, in recent unpublished studies we found that this combination exerts a synergistic inhibition of the growth of cholangiocarcinoma cells. These findings suggest the combination of cisplatin with Slug suppression might be an effective regimen for the chemoprevention and/or chemotherapy of various types of human malignancies.

## Figures and Tables

**Figure 1:** Slug regulation-induced processing of Slug and PUMA. (**A**) The protein fractions of Slug in QBC939, RBE, ICC-9810, and FRH 0201 cells were subjected to Western blot analysis. FRH 0201 exhibited the lowest expression level of Slug and QBC939 exhibited the highest expression level of Slug. (**B**) The protein fractions of Slug, E-cadherin, and PUMA in QBC939 cells after transfection with Slug siRNA for 48 h were subjected to Western blot analysis. Slug expression was barely detectable compared with parental cells (**P < 0.01), and a remarkble upregulation of E-cadherin and PUMA protein was shown compared with parental cells (*P < 0.05). (**C**) The protein fractions of Slug, E-cadherin, and PUMA in the FRH 0201 cell line after transfection with Slug cDNA for 48 h were subjected to Western blot analysis. Remarkable upregulation of Slug protein was shown compared with parental cells (**P < 0.01), and remarkable downregulation of PUMA and E-cadherin proteins was shown compared with parental cells (*P < 0.05).

**Figure 2:** TUNEL staining was performed for QBC939 cells transiently transfected with Slug siRNA or mock transfected for 48hs. Green nuclear staining indicates apoptotic cells. The percentage of TUNEL-positive cells was quantified. Columns and bars represent the mean and standard deviation of three independent determinations, respectively. Significant differences between the controls (mock) and the Slug siRNA groups are indicated by *P < 0.05.

**Figure 3:** Cisplatin-induced apoptosis in QBC939 and FRH 0201 cells. **A**, **C**, QBC939 and FRH0201 cells (1 × 10^6^/mL) were exposed to the designated concentrations of cisplatin for the indicated times, after which time the percentage of apoptotic cells was determined by flow cytometric analysis, as described in “Materials and Methods”. The data are expressed as a mean value of the percentage of apoptotic cells from three independent experiments performed in duplicate (*P < 0.05, **P < 0.01, ***P < 0.001). **B**, **D**, At the indicated time points after treatment with 20 μg/mL cisplatin, the cells were harvested and fixed in 70% ethanol. After staining with PI, the apoptotic DNA content was analyzed by flow cytometry. The number of apoptotic cells in the sub-G1 fraction is expressed as a percentage of the total number of cells (*P < 0.05, **P < 0.01, ***P < 0.001).

**Figure 4:** Induction of apoptosis by cisplatin is independent of PUMA mechanism. (**A**, **B**) The QBC939 and FRH 0201 cells were exposed to various cisplatin concentrations for 72 h. The PUMA and E-cadherin protein expression levels in the cell lysate were examined by Western blot analysis using anti-PUMA (E-cadherin) antibody, and the antibodies against ß-actin which served as an internal control. (**C**, **D**) The QBC939 and FRH 0201 cells were exposed to 20 μg/mL cisplatin for the indicated times. The PUMA and E-cadherin protein expression level was measured by Western blot. (**E**, **F**) QBC939 and FRH0201 cells (1 × 10^6^/mL) were exposed to 20 μg/mL cisplatin combined with PUMA siRNA for 72 h, PUMA protein expression level was measured by Western blot. (**G**, **H**) QBC939 and FRH0201 cells (1 × 10^6^/mL) were exposed to 20 μg/mL cisplatin combined with PUMA siRNA for 72 h, after which time the percentage of apoptotic cells was determined by flow cytometric analysis, as described in “Materials and Methods”. Cisplatin combined with PUMA siRNA did not induce obvious apoptosis in QBC939 and FRH 0201 cells (^*^P < 0.01).

**Figure 5:** TUNEL staining was performed to assess the potential cooperation of Slug silencing and cisplatin treatment in inducing apoptosis in QBC939 cells. Green nuclear staining indicates apoptotic cells. The percentage of TUNEL-positive cells was quantified. Columns and bars represent mean and standard deviation of three independent determinations, respectively. Significant differences between the controls (mock) and the Slug siRNA groups are indicated by *P < 0.05, **P < 0.01.

**Figure 6:** Slug silencing sensitizes cholangiocarcinoma xenograft tumors to cisplatin. **A**, growth bar of QBC939 tumors (n = 6 per group) subjected to Slug siRNA, mock, and PBS and/or combined with cisplatin treatment for 28 days. **B**, Immunohistochemistry analysis for Slug and PUMA in different groups. **C**, TUNEL-positive cells in three groups were detected in the control, cisplatin, or Slug siRNA plus cisplatin treatments. Columns and bars represent the mean of three independent determinations and S.D., respectively. *P < 0.05, **P < 0.01, ***P < 0.01.
